# Biogenic Synthesis of Silver Nanoparticles (AgNPs) Using Aqueous Leaf Extract of *Buchanania lanzan* Spreng and Evaluation of Their Antifungal Activity against Phytopathogenic Fungi

**DOI:** 10.1155/2022/6825150

**Published:** 2022-03-10

**Authors:** Ayushi Purohit, Radheshyam Sharma, R. Shiv Ramakrishnan, Stuti Sharma, Ashish Kumar, Devendra Jain, Himmat S. Kushwaha, Elina Maharjan

**Affiliations:** ^1^Jawaharlal Nehru Krishi Vishwa Vidyalaya, Jabalpur 482 004, India; ^2^Maharana Pratap University of Agriculture and Technology, Udaipur 313001, India; ^3^Malaviya National Institute of Technology, Jaipur 302017, India; ^4^Tribhuvan University, Kirtipur, Kathmandu, Nepal

## Abstract

Nanoparticles show the multidisciplinary versatile utility and are gaining the prime place in various fields, such as medicine, electronics, pharmaceuticals, electrical designing, cosmetics, food industries, and agriculture, due to their small size and large surface to volume ratio. Biogenic or green synthesis methods are environmentally friendly, economically feasible, rapid, free of organic solvents, and reliable over conventional methods. Plant extracts are of incredible potential in the biosynthesis of metal nanoparticles owing to their bountiful availability, stabilizing, and reducing ability. In the present study, the aqueous leaf extract of *Buchanania lanzan* Spreng was mixed with 0.5 mM silver nitrate and incubated at 70°C for 1 h and synthesized a good quantity of AgNPs. The synthesized AgNPs were characterized using UV-visible spectroscopy, X-ray diffractometry (XRD), dynamic light scattering (DLS), transmission electron microscopy (TEM), and scanning electron microscopy (SEM). The maximum absorption of UV-visible spectra was obtained in the range of 420–430 nm. Furthermore, SEM and TEM results inferred that the size of the particles were 23–62 nm, spherical, crystalline, uniformly distributed, and negatively charged with the zeta potential of −27.6 mV. In addition, the antifungal activities of the AgNPs were evaluated against two phytopathogenic fungi *Rhizoctonia solani* and *Fusarium oxysporum* f. sp. *lycopersici* in vitro using poison food techniques on PDA media. The maximum rate of mycelia inhibition was found in 150 ppm concentration of AgNPs against both phytopathogenic fungi.

## 1. Introduction

The field of nanotechnology is one of the zestful areas of research in modern material sciences and acquiring energy because of its capacity to change metals into nanoparticles. The nanotechnology field is growing steadily and creating an impact in all arenas of human life including agriculture, medicine, textiles, electronics, and pharmaceuticals [1]. Nanoparticles display totally novel and further developed properties dependent on explicit attributes such as size, dispersion, and morphology, typically groups of atoms in the size scope of 1–100 nm. Materials in nanodimensions have a notable difference in its physical and structural properties of atoms and molecules when compared to the similar material in mass due to the distinction in physicochemical properties and surface to volume ratio [2].

The antimicrobial properties of AgNPs have likewise been taken advantage of both in medicine and home. Because of their antibacterial properties, AgNPs have been utilized broadly in the wellbeing business, food stockpiling, material coatings, and numerous natural applications [3]. Conventionally, AgNPs are synthesized by the chemical technique utilizing synthetic compounds as reducing agents, which later on become responsible for different natural risks because of their overall harmfulness, inducing the genuine worry to foster climate cordial cycles [4]. The plant contains plentiful natural compounds such as alkaloids, flavonoids, saponins, steroids, tannins, and other nourishing mixtures. These natural compounds are derived from different parts of a plant like leaves, stem, roots, shoots, blossoms, barks, and seeds; these properties conjuring a new biosynthesis strategy is environment amicable since the plant extract contains different secondary metabolites and acts as reducing and stabilizing agents for the bioreduction reaction to synthesized novel metallic nanoparticles.

Plant extract is a cost-efficient, ecofriendly, and efficient substitute for the extensive synthesis of nanoparticles [5, 6]. In this perception, *Buchanania lanzan* Spreng (family: Anacardiaceae), an endemic perennial forest tree of India, commonly known as chironji, exhibits a striking assortment of shapes. The leaves of *B. lanzan* Spreng contain several secondary metabolites such as tannins, polyphenols, flavonoids, glycosides, saponins, triterpenoids, steroids, alkaloids, quercetin-3-rhamnoglucoside, kaempferol-7-O-glucosides, kaempferol, and myricetin 3′-rhamnoside-3-galactoside, analyzed though TLC and HPTLC techniques [7, 8]. Leaf juice of *B. lanzan* Spreng has high pharmaceutical value and commercially used to prepare several Ayurvedic and Unani medicines. Many Indian tribals are used for curing many disorders, joint pain, quick healing of wounds, purifying blood, treating loss of libido, impotency, augmenting the glow on the skin, and also as a tonic for the digestive system. These properties of *B. lanzan* can be helpful in reducing metallic salts into nanometallic particles. Hence, first time, *B. lanzan* Spreng leaf extract was used to produce a biodegradable nanosilver natural product without any risk of chemical toxicity. Characterizations of AgNPs are essential to check the functional aspects of the synthesized particles; their physicochemical properties include biodistribution, behavior, efficacy, and safety. Characterization was performed utilizing an assortment of scientific procedures, including X-ray diffractometry (XRD), UV-vis spectroscopy, dynamic light scattering (DLS), transmission electron microscopy (TEM), and scanning electron microscopy (SEM) [9–11].

There have been various efforts to manage plant diseases in the agro-ecosystem. Present, chemical control is widely applied which has several drawbacks, including the risk of toxicity, stability, and environmental hazards. Therefore, present need is to identify eco-safe, cost-effective, and target specific with greater biocompatibility of biomolecules to control the plant pathogens. Green-synthesized AgNP is an effective antimicrobial agent against diverse range of plant pathogens and emerging as novel and economical technology [12]. AgNPs exerted intense antifungal impact on fungi growth tested in vitro, most likely through annihilation of membrane integrity [13]. Because of their size, AgNPs can enter cells, hinder enzymatic frameworks in the respiratory chain of certain microorganisms, and in this way, alter their DNA synthesis. The suspension of AgNPs showed antibacterial action against the reference strain and on hospital strains that were impervious to most of the antibiotics [14]. The ability of AgNPs to bind on fungal cell wall and membrane and produce reactive oxygen species and free radicals activates cellular toxicity and oxidative stress and regulation of the signal transduction pathway. It is therefore anxious to evaluate the antifungal effect of synthesized AgNPs against phytopathogenic fungi, which can be utilized in the field of nanotechnology as a cost-effective, ecofriendly, and green strategy. Hence, first time, AgNPs were synthesized using *B. lanzan* Spreng and assesses their antimicrobial activity against phytopathogenic fungi.

## 2. Materials and Methods

### 2.1. Plant Material and Preparation of the Extract

For the preparation of the plant extract, approximately 5 g of sterilized green leaves of *B. lanzan* Spreng was taken, chopped, and put in a beaker with 100 ml distilled water and boiled on a hot plate for 5 min. Furthermore, the boiled solution was allowed to cool at room temperature and filtered by Whatman filter paper no. 1.

### 2.2. Preparation of AgNO_3_ Solution and Green Synthesis of the AgNPs

The plant extract was mixed with 0.5 mM silver nitrate in 5% by volume ratio, and the reaction mixture was incubated in the amber jar for 1 h at 70°C temperature for reduction of Ag + ions. A change in the colour of the solution was observed from transparent to brown, with a pungent smell after incubation, indicating the formation of AgNP by the reduction of AgNO_3_. After completion reduction, AgNPs were purified by repeated centrifugation at 10000 rpm for 10 min. The obtained pellet was redispersed in deionized water, and the sample was stored at room temperature in dark.

### 2.3. Characterization of AgNPs

#### 2.3.1. UV-Visible Spectroscopy (UV-Vis Spectral) Analysis

The reduction of pure Ag^+^ ions to AgNPs was checked by estimating the UV-vis range of the response medium from 30 min–5 hours. UV-vis spectral examination was done by utilizing the nanophotometer (Genova, UK), and the absorbance was recorded at a frequency range of 300–600 nm.

#### 2.3.2. X-Ray Diffraction (XRD) Analysis

The liquid solution of AgNPs was centrifuged repeatedly and dried in a lyophilizer (New Brunswick Scientific, USA). Furthermore, the composition and structure of purified AgNPs were analyzed by an X'Pert Pro X-ray diffractometer (PAN analytical BV, the Netherlands) run at a voltage of 45 kV and an electric power of 35 mA with Cu K*α* radiation in *θ*–2*θ* configuration. The crystallite space size was determined from the width of the XRD peaks, expecting that they are free from nonuniform strains, using the Scherrer formula:

(1) $$\begin{array}{c} D=\frac{0.94\;\lambda }{\beta \;\cos\;\theta }, \end{array}$$

where *D* is the normal crystallite domain size opposite to the reflecting plane, *λ* is the X-ray wavelength, *β* is the full width at half most extreme (FWHM), and *θ* is the diffraction point. To wipe out extra instrumental widening, the FWHM was rectified, utilizing FWHM from a substantial grained Si sample.

(2) $$\begin{array}{c} \beta \text{ corrected }={\left({\text{FWHM}}_{\text{sample}}^{2}-{\text{FWHM}}_{si}^{2}\right)}^{1/2}. \end{array}$$

This modified formula is legitimate just when the crystallite size is < 100 nm.

#### 2.3.3. Scanning Electron Microscope (SEM) Analysis

On a carbon-coated copper framework, thin films of the sample were prepared by simply just dropping a very small amount of the sample on the grid, and then, the film on the SEM grid was permitted to dry by putting it under a mercury lamp light for 5 min. EDS estimations of the *B. lanzan* Spreng reduced AgNPs drop coated onto Si (111) wafers were executed on a Leica Stereoscan 440 SEM instrument equipped with a Phoenix EDAX attachment.

#### 2.3.4. Transmission Electron Microscopy (TEM) Analysis

For TEM analysis, samples were prepared on a carbon-coated copper TEM grid on the Joel JEM1400 TEM machine. The films on the TEM grid were permitted to locate for 2 min, following which the additional AgNPs sample was detached using a blotting paper, and the grid was permitted to dry under an infrared lamp before measurement. The clear spots in the SAED pattern showed the crystalline nature of AgNPs.

#### 2.3.5. Dynamic Light Scattering (DLS) and Zeta Potential Analysis

Zeta potential and size distribution of AgNPs were determined by dynamic light scattering (DLS) using Malvern Zetasizer Nano series (UK), and analysis was accomplished for sizes ranging from 0.1 nm to 10 *µ*m.

### 2.4. Evaluation of Antifungal Activity of AgNPs against Phytopathogenic Fungi

The efficacy of AgNPs against fruit rot (*Rhizoctonia solanum*) and wilt (*Fusarium oxysporum* f. sp. *lycopersici*) of tomato strains was assessed using the poison food technique [9] by supplementing the potato dextrose agar (PDA) media (HiMedia, India) with 50 ppm, 100 ppm, and 150 ppm of the final concentration of dried lyophilized AgNPs samples. The agar plugs of uniform size (diameter, 5 mm) were picked using a sterilized cork borer from the Petri dish having full growth of phytopathogenic fungi and inoculated at the middle of every Petri dish (90 mm) containing AgNPs and kept at 25 ± 2°C for 5 days. After incubation of fungi on the PDA medium containing AgNPs, radial growth of fungal mycelium was observed and accompanying equation was utilized for the computation of the inhibition rate (%).

(3) $$\begin{array}{c} \text{Inhibition rate }\left(\%\right)=\left(\frac{R-r}{R}\right)\times 100, \end{array}$$

where “*R*” is the radial growth of fungal mycelia on the control Petri dish; whereas, “*r*” is the radial growth of fungal mycelia on the Petri dish treated with AgNPs.

### 2.5. Statistical Analysis

The obtained results of the in vitro antifungal assay were subjected to statistical analysis. Moreover, for determining significant differences among variable treatments on various AgNPs, the analysis has been done using JMP software version 11 (SAS, 2009) utilizing the Turkey–Kramer HSD *t*-test, *p*=0.05.

## 3. Results and Discussion

### 3.1. Synthesis of AgNPs Using Leaf Extract of *B. lanzan* Spreng

In the present time, biogenic methods of reducing metals are gaining tremendous impetus in the field of nanotechnology. In the present study, *B. lanzan* Spreng leaf extract was employed for the synthesis of AgNPs. *B. lanzan* Spreng is an Indian native forest tree species and have tremendous application in the pharmaceutical industry and Indian medicine system (IMS). Initially, several synthesis parameters such as pH, temperature, incubation time, and concentration of AgNPs were standardized. For standardization of synthesis parameters, the leaf extract of *B. lanzan* Spreng was blended with different concentrations of silver particle complex solution and incubated. After incubation, it starts to begin changing the colour from watery to brown with a pungent smell owing to the reduction of silver to silver ions by electron donor metabolites present in the leaf extract, which is the primary apparent indication of AgNPs synthesis. Furthermore, by keeping one parameter stable at a time, the proportion of the intensity of colour changes was monitored and standardized all parameters. The reaction mixture containing AgNPs was monitored under the UV-vis spectrophotometer, and the highest absorbance could be recorded at 420–430 nm (Figure 1). Analysis at different temperature regimes, viz., 40–70°C and incubation period (1–5 h) revealed the maximum synthesis of AgNPs at 70°C temperature after one hour of incubation. Finally, after standardizing all parameters, 0.5 mm silver nitrate was added to aqueous leaf extract of *B. lanzan* Spreng in an amber flask and incubated at 70°C for 1 h synthesis yielded good quality and quantity of AgNPs. In this way, incubation for one hour at 70°C temperature could be standardized for successful synthesis of AgNPs. Previously, Jain et al. [15] synthesized AgNPs using aqueous leaf extract of *Tagetes patula* and obtained good quality nanoparticles.

### 3.2. Characterization of Synthesized AgNPs Using XRD and TEM Analyses

The synthesized AgNPs were characterized by XRD and TEM. Structure and crystalline nature of synthesized AgNPs were executed by XRD and showed peaks at 2*θ* = 38°, 45°, 65°, 78°, with the highest intensity at 2*θ* = 38° (Figure 2). The present results were corroborated by Mehta et al. [7] and Abdulwahid et al. [16]. They found it to be 2*θ* = 40; by comparing this, the presence of AgNPs can be confirmed in the sample. Latha et al. [17] suggested that the structure of AgNPs is FCC and crystalline in nature.

TEM analysis of the AgNPs synthesized using aqueous extract confirmed their size, shape, and distribution. The size of the particles was 14.09 nm, and the shape varied from oval to spherical with a narrow size distribution (Figures 3(a) and 3(b)). Similar to our previous results, Sun et al. [18] and Su et al. [19] inferred the spherical shape of AgNPs by TEM.

### 3.3. Characterization of AgNPs Using Scanning Electron Microscope (SEM) and Energy Dispersive X-Ray (EDX)

The characterization of particle size, nanomaterial shape, size distributions, and surface morphology of the synthesized particles at microlevel and nanolevel were performed using SEM. The particle size varied from 25.95 nm to 65.10 nm with uniform distribution of particles. The microscopy was done in different magnification scales, and the shape of the particles was inferred to be spherical (Figures 4(a)–4(d)). The resulting aggregates were dense and also exhibited fractal shapes, which may be attributed due to uninterrupted crystalline packing of ligands on particle surfaces. Energy dispersive X-ray (EDX) of the AgNP drop coated on Si (III) wafers was performed for revealing the presence of AgNP and other elements present in the sample. EXD graph results showed that no other elemental impurity was present in the synthesized AgNPs, and only a trace amount of oxygen could be detected (Figure 5). Earlier, a study conducted by Dhand et al. [5] conquered the presence of polymorphic shapes such as flake type, rocky, spherical, ellipsoidal, and irregular granulated compact/fused agglomerates of powder with brighter facets. They likewise observed that each agglomerate is melded freely at their ends. The normal sizes of these agglomerates were in the scope of 3 *μ*m–20 *μ*m, respectively.

### 3.4. Characterization of AgNPs Using Zeta Potential Analysis

The DLS analysis was observed by analyzing the zeta potential of the synthesized AgNPs, and the result revealed that polydispersivity index (PDI) was very less as a single peak is formed, so we can infer the uniformity of particles in a dispersive medium. The value of zeta potential was −27.6, indicating that the sample was highly stable; as generally a sample with value ± 30 mV is considered a stable sample, the negative sign indicates that it is negatively charged, and also, the mean area of the single peak is 99.7%, which indicates a uniform negative charge between the particles in the polydispersive medium. The conductivity of the sample was low, as depicted by the graph (Figure 6). Previously, Chaudhuri et al. [20] also synthesized AgNPs from leaf extract of *Tecomella undulata* and found the zeta potential was −16 with two peaks.

### 3.5. Assessment of Antifungal Activity of AgNPs against Phytopathogenic Fungi

The antifungal activity against *Rhizoctonia solani* was evaluated by the poison food technique using the PDA medium. At 150 ppm concentration of AgNPs, the maximum percent inhibition of 52.16% in the mycelial growth of *Rhizoctonia solani* was observed after 5 days of incubation. However, minimum inhibition was recorded at 50 ppm concentration (Table 1). There was clear inhibition in growth of *R. solani* at all the tested concentrations of AgNPs in comparison to control which indicated the possible use of AgNPs in controlling this multiphagous pathogen after successful evaluation under in vitro conditions (Figure 7).

In *Fusarium oxysporum* f. sp. *lycopersici*, 47.08% inhibition of mycelia growth was observed at 150 ppm concentration of AgNPs after 05 days of inoculation (Table 2). The radial growth of the fungus on the PDA medium and their zone of inhibition are depicted (Figure 8). Earlier, Sukhwal et al. [21] also studied the antifungal activity of AgNPs by the poison food technique on PDA media using phytopathogenic fungi *Colletotrichum chlorophyti* and obtained the maximum percent inhibition at 100 ppm concentration of AgNPs. In the present investigation, antifungal activity of AgNPs has been proven against two major soilborne fungal pathogens of chickpea, opening the avenues for exploiting the use of nanoparticles in plant disease control.

## 4. Conclusion

Recently, plant extracts have become attractive methods for the reduction of ions, and they act as reducing and capping agents. *B. lanzan* Spreng, an endemic forest plant species of India, contains several essential secondary metabolites and has the potential to reduce AgNO_3_ into AgNPs. Taking into consideration the various advantages of green synthesis of AgNPs and the use of plant extracts and their top-notch antimicrobial activities, there is no doubt that this research field will continue to attract an awful lot interest in current years. The *B. lanzan* Spreng containing AgNPs was assessed under the UV-vis spectrophotometer, and the highest absorbance was obtained at 406 nm. XRD results revealed the presence of silver in the sample. SEM results reveal the spherical shape and size of AgNPs, which varied from 25.09 nm to 65.25 nm, and the average size of the particles was 42.3 nm. Moreover, the EDX results revealed the absence of contamination in the sample. Only oxygen was present in a very trace amounts other than silver. TEM results reveal the oval to spherical shape of the sample, and the size was found to be 14.09 nm, and also, the reports reveal the crystalline nature of AgNPs. The zeta potential was found to be −27 Mv by DLS results, and the results reveal that the sample is stable, uniform, has low conductivity, and was negatively charged. The antifungal activity of AgNPs against *Rhizoctonia solanum* and *Fusarium oxysporum* f. sp. *lycopersici* was evaluated and obtained the maximum percent of mycelia growth inhibition at 150 ppm concentration in fungi. This study presents valuable information concerning the antimicrobial and phytopathogenic efficacies of *B. lanzan* Spreng leaf extract-mediated AgNPs. The nanoparticles may be similarly subjected to toxicity assays, and further research needs to be designed in order to assess the effects, so they could produce to soil, plants, and environment, in general, due to long-term exposure. Therefore, local and countrywide regulatory institutions must set up guidelines and monitoring strategies for better use of these nanotechnological advances.

## Figures and Tables

**Figure 1:** UV-vis absorption spectra of AgNPs using *B. lanzan* Spreng leaf extract.

**Figure 2:** XRD analysis of AgNPs synthesized using *B. lanzan* Spreng leaf extract.

**Figure 3:** (a) TEM micrograph and (b) SEAD pattern of AgNPs synthesized using *B. lanzan* Spreng.

**Figure 4:** (a)–(d) SEM micrograph of AgNPs synthesized using *B. lanzan* Spreng leaf extract at different magnification scales.

**Figure 5:** EDX graph of AgNPs synthesized using *B. lanzan* Spreng leaf extract.

**Figure 6:** (a) Size distribution. (b) Zeta potential distribution of AgNPs synthesized using *B. lanzan* Spreng leaf extract.

**Figure 7:** Antifungal bioassay of AgNPs against *Rhizoctonia solani* by the poisoned food technique. (a) 150 ppm. (b) 100 ppm. (c) 50 ppm. (d) Control. The observation was recorded after 7 days of incubation.

**Figure 8:** Antifungal bioassay of AgNPs against *Fusarium oxysporum* by the poisoned food technique. (a) 150 ppm. (b) 100 ppm. (c) 50 ppm. (d) Control. The observation was recorded after 3 days of incubation.

**Table 1:** Antifungal activity of AgNPs on in vitro mycelial growth of *Rhizoctonia solani*.

Treatment	% inhibition mycelia growth^a^
Control^b^	0.0^D^
50 ppm	47.22 ± 0.82^C^
100 ppm	52.16 ± 0.76^B^
150 ppm	75.01 ± 0.876^A^

^a^Each value is the mean of the three replicates. Mean ± SE followed by the same letter in the column of each treatment represents no significant difference at *p*=0.05 by the Tukey–Kramer HSD test. % inhibition rate was calculated compared with mycelial growth of the control (0%). ^b^Control without any formulation. The observations were recorded after 5 days of incubation.

**Table 2:** Antifungal activity of AgNPs on in vitro mycelial growth of *Fusarium oxysporum* f. sp. *lycopersici*.

Treatment	% inhibition mycelia growth^a^
Control^b^	0.0^D^
50 ppm	9.09 ± 0.65^C^
100 ppm	20.70 ± 0.14^B^
150 ppm	47.08 ± 0.67^A^

^a^Each value is the mean of the three replicates. Mean ± SE followed by the same letter in the column of each treatment represents no significant difference at *p*=0.05 by the Tukey–Kramer HSD test. % inhibition rate was calculated compared with mycelial growth of the control (0%). ^b^Control without any formulation. The observations were recorded after 5 days of incubation.

## Data Availability

The data generated during this study are available at Biotechnology Centre, Jawaharlal Nehru Krishi Vishwa Vidyalaya, Jabalpur 482004, India, and are available from the corresponding author upon request.
